# What Does It Cost to Prevent On-Duty Firefighter Cardiac Events? A Content Valid Method for Calculating Costs

**DOI:** 10.1155/2013/972724

**Published:** 2013-12-22

**Authors:** P. Daniel Patterson, Joe Suyama, Steven E. Reis, Matthew D. Weaver, David Hostler

**Affiliations:** University of Pittsburgh School of Medicine, Department of Emergency Medicine, 3600 Forbes Avenue, Suite 400A, Pittsburgh, PA 15261, USA

## Abstract

Cardiac arrest is a leading cause of mortality among firefighters. We sought to develop a valid method for determining the costs of a workplace prevention program for firefighters. In 2012, we developed a draft framework using human resource accounting and in-depth interviews with experts in the firefighting and insurance industries. The interviews produced a draft cost model with 6 components and 26 subcomponents. In 2013, we randomly sampled 100 fire chiefs out of >7,400 affiliated with the International Association of Fire Chiefs. We used the Content Validity Index (CVI) to identify the content valid components of the draft cost model. This was accomplished by having fire chiefs rate the relevancy of cost components using a 4-point Likert scale (highly relevant to not relevant). We received complete survey data from 65 fire chiefs (65% response rate). We retained 5 components and 21 subcomponents based on CVI scores ≥0.70. The five main components include, (1) investment costs, (2) orientation and training costs, (3) medical and pharmaceutical costs, (4) education and continuing education costs, and (5) maintenance costs. Data from a diverse sample of fire chiefs has produced a content valid method for calculating the cost of a prevention program among firefighters.

## 1. Introduction

Firefighters in the United States suffer cardiac-related line of duty death (LODD) at exceedingly high rates with events 10–100 times more likely to occur during, or in the hours immediately following, fire suppression [1]. The underlying mechanism for cardiovascular events among firefighters is unknown, but it is believed to be multifactorial including both occupational and lifestyle factors. Occupational factors such as shift work, lifestyle factors, and the exposures associated with fire suppression (e.g., smoke, chemicals) may predispose the firefighter to earlier onset of heart disease [2]. Additionally, rates of hypertension, overweight, and obesity within the fire service exceed those seen in the general population increasing the baseline risk for a cardiovascular event [3, 4].

Fire suppression activities result in significant cardiovascular strain and provide potential triggers for ischemic events (e.g., myocardial infarction, stroke). There is a rapid rise in heart rate following the activation of a fire department which may persist for as long as 20 minutes [5, 6]. Even in cases where heavy work is not being performed, the repetitive upper body exercise associated with tool use raises heart rate disproportionately to oxygen consumption [7]. Finally, the heat stress associated with fire suppression has been shown to enhance coagulation potential and activate platelets reducing platelet closure time [8–10].

Given the multiple risk factors and potential triggers for cardiovascular events associated with fire suppression, there is a tangible need for preventative measures among firefighters. Potential interventions include weight loss and fitness programming initiatives and pharmaceutical interventions. Two studies have been funded through the FEMA Fire Prevention & Safety mechanism to examine the role of daily or acute aspirin on platelet activation in firefighters. However, the cost and benefit for these types of programs have not been examined in great detail within the fire service. Lack of a valid method for quantifying costs with any type of intervention, fitness or pharmacological, may prevent program adoption amongst those most likely to benefit from a prevention program. In this study, we sought to create a valid method for quantifying the costs of programs that aim to reduce firefighter mortality related to on-duty cardiac events.

## 2. Methods

We used a mixed-method approach approved by the University of Pittsburgh Institutional Review Board that included qualitative in-depth interviews, a cross-sectional survey, and validity calculation. First, in 2012, we performed in-depth interviews with four experts. The experts included a convenience sample of fire department chiefs, mid-level department administrators, and a representative of insurance companies. We included a representative from the insurance industry in order to identify the principal components of cost that an insurance company might cover for a fire department. We recruited these experts from a convenience sample of experts listed in an internally maintained database of fire industry contacts who have participated in previous fire safety research.

Our in-depth interviews were guided by theories of costs estimation accepted in Human Resource Accounting (HRA), which includes direct and indirect costs [11]. Direct costs refer to materials, goods, and other tangibles commonly listed on balance sheets and budgets as reoccurring or one-time purchases with capital from the organization. Indirect costs refer to the time that organizational staff devotes to specific components of their occupation. We chose to follow a HRA framework based on evidence of “real world” utility and application of previously developed HRA-based cost models [12–16]. We used HRA to frame our interview questions, which were designed to identify common themes/components of costs considered important and relevant by industry experts. For example, we asked expert interviewees to consider and comment on the amount of time employees may devote to activities such as exercising and continuing education while on-duty and the costs that a fire department may incur as a result. This is an example of indirect costs [12–16]. We ended in-depth interviews once the interviewer declared saturation [17]. Saturation refers to the point when the interviewer determines that interviewees are no longer expanding the range of information on a cost component or offering new information beyond that already provided.

Next, in 2013, we randomly sampled 100 fire chiefs from the International Association of Fire Chiefs (IAFC) database of 7,461 fire chiefs located within the USA and internationally. We then contacted each fire chief via a mailed recruitment packet. The packet included (1) a description of the study, (2) letter of support from the National Fallen Firefighters Foundation (NFFF), and (3) a $5.00 gift card. The recruitment letter directed fire chiefs to a study web site where they rated the relevancy of each component of the draft method for calculating costs. We obtained ratings with a four-point Likert scale anchored from “Highly Relevant” to “Not Relevant.”

Finally, we calculated the content validity of fire chief ratings using the widely accepted Content Validity Index (CVI). The CVI is proportion of raters assigning a rating of 3 = *quite relevant* or 4 = *highly relevant* [18]. Two CVI scores may be calculated, one for components (the Scale-CVI or S-CVI) and one for subcomponents (the Item-CVI or I-CVI) [18]. We calculated S-CVI and I-CVI scores based on techniques developed by Lynn, Waltz, and Bausell with S-CVI and I-CVI scores ≥0.70 as benchmarks for content validity in this study [18]. We then stratified subcomponents into direct and indirect costs.

## 3. Results

In-depth interviews with our four experts resulted in a draft method for cost calculation that included six components and 26 subcomponents. Components included (1) preparatory costs, (2) investment costs, (3) orientation and training costs, (4) medical care and pharmaceutical costs, (5) education and continuing education costs, and (6) maintenance costs.  Figure 1 is a graphical illustration of this draft model for cost calculation.

We received 65 completed surveys from fire chiefs (65% response rate). The S-CVI score for preparatory costs (0.66) fell below the 0.70 benchmark suggesting that fire chiefs do not believe this component should be considered a valid part of cost calculation (Table 1). Content validity scores showed that two additional subcomponents fell below the 0.70 cut point for I-CVI. These include one subcomponent of direct costs for the Orientation & Training Costs component and one subcomponent of Education & Continuing Education component.

In total, greater than 70% of fire chiefs surveyed in this study found five of the original six components of costs and 21 of the original 26 subcomponents to be content valid. CVI scores were highest (quite relevant to highly relevant) for the medical and pharmaceutical Costs component, suggesting most fire chiefs were supportive of this component and its subcomponents.  Table 2 presents a final draft of the method for calculating costs of a firefighter program to reduce on-duty related cardiac events.

## 4. Discussion

Risk of morbidity and mortality from cardiovascular events in the line of duty is high among firefighters [1]. Fire chiefs, fire department insurers, and others share a common concern for firefighter health, wellness, and safety. There are numerous potential solutions for reducing risk; however, the costs associated with these solutions or programs are unknown and likely vary by fire department. We have developed a model to aide fire chiefs that can support the calculation of cost associated with the implementation and maintenance of a program to prevent cardiovascular events or reduce the cardiovascular-related morbidity and mortality among firefighters. Our model represents a starting point from which fire chiefs and others can begin. Application of this model to a candidate program or intervention is required to fully test model efficacy. Lack of data from any actual model application precludes us from evaluating select measures of reliability, construct validity, and predictive validity. The principal benefit of this model is its validity. The components and subcomponents of this model were developed based on a widely accepted framework for cost estimation and calibrated to fit the fire industry with input from 65 randomly sampled fire chiefs.

Like those before us [12–16], we began by developing a framework for cost calculation based on the Human Resource Accounting (HRA) approach. We have demonstrated success with this approach in the past by developing a model for determining the cost associated with turnover in Emergency Medical Services (EMS) organizations [19]. Others have applied the HRA approach as well, which we believe is supportive evidence for HRA's value in development of cost calculation modeling [12–16]. However, we believe that no one approach is optimal and acknowledge that additional research is needed to: (1) fully expose known and unknown factors associated with program cost using different frameworks, (2) to determine feasibility in application in organizations to which they were designed; and (3) to document the perceived utility among the administrators that will use these models.

The value of our work at this time is supported by the growing body of evidence that cardiovascular events are the most common cause of firefighter line-of-duty death and believed to be higher than other professions [1]. We have previously shown that, in one large community, non-fatal cardiac events occur in similar proportions for fire, police, and EMS making this tool widely applicable across public safety [20]. Improving firefighter fitness is a key step in reducing the number of job-related cardiovascular events [21]. However, there are exposures and stressors associated with fire suppression that cannot be mitigated by fitness alone [2]. Therefore, it is reasonable for the fire service to pursue both fitness related programs and other potential solutions such as technology (e.g., physiologic monitoring, enhanced respiratory protection) and pharmacotherapy to reduce the number of cardiovascular events in public safety providers.

Our work will also help expedite future work employing cost-benefit, cost-effectiveness, and related types of economic valuation and analysis techniques. These techniques require multiple steps, including the identification and gathering of data to value costs of diverse decision options [22]. Experts in methods for quantitative synthesis point out that the single most common thread among all techniques is cost valuation or the determination of costs [22]. Given its importance, the overarching goal of cost-effectiveness analysis—to compare the outcome of different decision options in terms of their costs—is not achievable without a comprehensive identification of costs, including direct and indirect costs [22]. In this study, we have demonstrated a focused effort to comprehensively identify the contributors to the cost of a prevention program for firefighters. Our study has addressed a gap not yet filled by the literature and completed a fundamental step to cost analyses that will accelerate future efforts to reduce firefighter morbidity and mortality.

We recognize that many recommendations exist for improving firefighter health and safety. Reports in the peer-reviewed literature have examined the utility of standard health surveillance [23], advanced imaging [24–26], and the potential need for enhanced respiratory protection following fire suppression [27, 28] to mitigate the risk of cardiovascular disease among firefighters. However, few studies have examined the costs associated with these programs [24]. Additionally, there are two trials of aspirin therapy in firefighters to reduce heat stress-induced platelet activation (http://www.clinicaltrials.gov). It is likely that a clinically viable program will be identified to improve the health and safety of the public safety provider. However, given limited resources in a public safety organization, the costs associated with new programs must be balanced against the existing operations' needs of that organization.

## 5. Limitations

Our study was limited by the sample of key informants, experts, and stakeholders interviewed and the 65 fire chiefs that responded to our survey. There is reason to believe that additional elements costs may have surfaced with added interviews and responses from additional fire chiefs. However, our sample was selected at random and more than half of fire chiefs surveyed provided input on the relevancy (content validity) of the method for cost calculation.

## 6. Conclusions

The cost calculation model presented in this paper represents formative work towards calculating the costs associated with programs and interventions led by fire department administrators targeting firefighters. We believe this model is a starting point for prevention in a higher risk industry and has broad applicability for industries with low penetration of prevention programs. While formative, decision makers may use this model as a framework for determining cost of prevention programs.

## Figures and Tables

**Figure 1:** Basic model for cost calculation.

**Table 1:** Content validity scores for each draft component (direct and indirect) of the method for calculating costs.

Component	Subcomponents used to operationalize direct and indirect elements of cost		Scale-CVI	Item-CVI
Preparatory costs	Direct	In the 3 months prior to adopting your program, record the amount of organizational capital disbursed to the following: (a) resource documents such as articles and text on cardiovascular disease among firefighters ($$$);	**0.66**	0.74
		(b) meetings and seminars ($$$);		0.74
		(c) travel to meetings and seminars concerned with cardiovascular disease among firefighters ($$$);		**0.57**
		(d) other resources that provided you with background information and guidance on addressing cardiovascular disease and death among firefighters ($$$).		**0.65**
	Indirect	In the 3 months prior to adopting your program, record the number of hours devoted to researching/investigating the program. Record these hours for each individual employed by the company: i.e., fire chief = (HH:MM); deputy chief = (HH:MM); shift supervisor = (HH:MM); other = (HH:MM).**		**0.62**

Investment costs	Direct	Consider 3 months prior and 1 month after program adoption and record the amount of organizational capital disbursed to a company or companies licensing the program ($$$).	0.77	0.82
	Indirect	Record these hours for each individual employed by the company devoted to communicating with program officials via meetings, telephone calls, and other communication: i.e., fire chief = (HH:MM); deputy chief = (HH:MM); shift supervisor = (HH:MM); other = (HH:MM).**		0.72

Orientation and training costs	Direct	In reference to each month after program adoption, record the amount of organizational capital disbursed to the following: (a) program manuals and materials such as pamphlets ($$$);	0.73	0.72
		(b) costs for copying materials for handouts to employees ($$$);		**0.52**
		(c) payment to speakers/guest speakers/medical personnel/trainers paid to provide guidance on program processes and/or training to employees ($$$).		0.83
	Indirect	In reference to each month after program adoption, record the hours for each individual employed by the company devoted to scheduling orientation and training, including time spent preparing materials and time spent communicating with program officials: i.e., fire chief = (HH:MM); deputy chief = (HH:MM); shift supervisor = (HH:MM); other = (HH:MM).**		0.75
		Record the amount of time that each employee participating in the program devoted to orientation and training while being “on the clock” at the fire station (HH:MM).**		0.74
		Record the amount of overtime (or unscheduled/additional) worked by employees covering for their colleagues while they attend orientation and training (HH:MM).**		0.74

Medical and pharmaceutical costs	Direct	In reference to each month after program adoption, record the amount of organizational capital disbursed to the following: (a) health physicals for employees ($$$);	0.82	0.88
		(b) medical tests not included in physical exams such as reoccurring visits to phlebotomists for laboratory tests ($$$);		0.88
		(c) payment for pharmaceuticals not covered by employee insurance programs ($$$);		0.86
	Indirect	In reference to each month after program adoption, record the hours each individual employed by the company devoted to visiting their physician/provider for a physical while being “on the clock” (HH:MM).**		0.79
		Record the amount of time that each employee devoted to medical tests not included in physical exams such as reoccurring visits to phlebotomists for laboratory tests—while being “on the clock” ($$$).**		0.74
		Record the amount of overtime (or unscheduled/additional) worked by employees covering for their colleagues while they completed the tasks listed as direct costs for this component (HH:MM).**		0.75

Education and continuing education	Direct	In reference to each month after program adoption, record the amount of organizational capital disbursed to the following: (a) supporting travel and expenses for employees to attend meetings/seminars/conferences related to the program's mission ($$$);	0.74	0.75
		(b) educating and training new hires on program requirements and parameters ($$$);		**0.68**
		(c) payment for speakers and materials that provide ongoing/focused education or continuing education on components of the program—outside of (in addition to) an existing continuing education program supported by the organization ($$$).		0.79
	Indirect	In reference to each month after program adoption, record the hours each individual employed by the company devoted to visiting education and continuing education linked to the program and while being “on the clock” (HH:MM).**	0.71	0.71
		Record the amount of overtime (or unscheduled/additional) worked by employees covering for their colleagues while they completed the tasks listed as direct costs for this component (HH:MM).**		0.71

Maintenance costs	Direct	In reference to each month after program adoption, record the amount of organizational capital disbursed to the following: (a) travel and expenses associated with company administrators (e.g., chiefs, deputy chiefs, etc.) devoted to attending meetings, seminars, conferences, and other events that provide ongoing instruction on program implementation and management ($$$). These expenses should be outside of (in addition to) costs accounted for in other cost components.	0.77	0.77
	Indirect	In reference to each month after program adoption, record the hours company administrators devoted to the direct costs activities while being “on the clock” for the organization (HH:MM).** If paid by the hour, record the amount of overtime (or unscheduled/additional) worked by administrators (HH:MM).**	0.72	0.72

Table notes: Components and subcomponents colored in bold font fail to meet the 0.70 cut-point/benchmark for content validity in this study and thus should be removed from the final algorithm, which is presented in Table 2.

**The algorithm will require multiplying hours (time) by the hourly rate per person. Apply the hourly wage for employees paid per hour. For salaried personnel, divide the salary by a standard work year (50 weeks) and workweek (37–40 hours) to determine hourly wage for cost calculation.

**Table 2:** Detailed description (example application) of the method for cost calculation.

The summation of direct cost components (Formula 1) can be used as a crude formula for calculating direct cost, unadjusted for total months. *Formula 1: y* = *ICDC* + *OTCDC* + *MPCDC* + *ECEDC* + *MCDC*. Where IC: investment costs, OTC: orientation and training costs, MPC: medical and pharmaceutical costs, ECE: educational and continuing education costs, and MC: maintenance costs.	
Formula 2 can be used to calculate time-adjusted direct cost biannually and annually. *Formula 2: y* = *ICDC*∑*h* + *OTCDC*∑*h* + *MPCDC*∑*h* + *ECEDC*∑*h* + *MCDC*∑*h*	
Where ∑*h* is the specified sum of months (i.e., 6 months, 12 months)	
Formula 3 excludes investment direct costs [*ICDC*∑*h* ] unique to the first year of program adoption and implementation and is adjusted for biannual and annual calculations. *Formula 3: y* = *TCDC*∑*h* + *MPCDC*∑*h* + *ECEDC*∑*h* + *MCDC*∑*h*	
For each component (IC, OTC, MPC, ECE, and MC), the direct costs may be found in administrative expense records. Quantifying indirect costs requires additional calculations where the hourly wage (or hourly equivalent for salaried personnel) is multiplied by the hours of the employees that devoted time to one or more components of the program. For example, a fire chief may document 20 total hours of his/her time to the OTC component during the third month of program implementation. To calculate indirect costs, the chief's hourly wage is needed. With an annual salary of $75,000, the chief's hourly wage would equal $41.21 dollars based on the definition of a full-time equivalent workweek of ≥35 hours per week	
[$41.21 per hr = ($75,000.00 annual salary)/(35 hrs per wk (52 weeks per year) = 1,820 hrs)].	
With these data, the estimated total indirect costs for OTC in month 3 would be $824.20.	
The example above should be replicated for all staff members that engage in activities or tasks linked to any of the six components of program costs (See Table 1). In other words, quantifying indirect costs should not be limited to administrative personnel and should include line-staff workers (front-line workers) who devote time to the program. Failure to consider these indirect costs would produce an underestimation of total program costs to the department/agency.	
Formula 4 is an example calculation model for quantifying indirect costs linked to time devoted to orientation and training. *Formula 4:* [*OTCID* = ∑_*i*−*j*_(*hrs*∗*wage*)]. Where OTCID indicates “indirect costs” and ∑_*i*−*j*_(*hrs*∗*wage*) is the product of hours of work devoted to OTC and hourly wage summed for all staff members[∑_*i*−*j*_] that devoted time to OTC related activities and tasks.	
Formula 5 can be used to quantify the total cost of the program adjusted for time, direct, and indirect costs. *Formula 5: y* = *ICDC* + *ID*∑*h* + *OTCDC* + *ID*∑*h* + *MPCDC* + *ID*∑*h* + *ECEDC* + *ID*∑*h* + *MCDC* + *ID*∑*h*	
Where *y* is the total program cost adjusted for time, direct, and indirect costs. Investment costs [*ICDC* + *ID*∑*h*] should be included for the first year calculation but removed in subsequent years.	
